The article "Application of the LINEX Loss Function with a Fundamental Derivation of Liu Estimator" was published in 2022. Journal: Comput Intell Neurosci.

# Application of the LINEX Loss Function with a Fundamental Derivation of Liu Estimator

**DOI:** 10.1155/2022/2307911

**Published:** 2022-03-14

**Authors:** M. A. Mohammed, Huda M. Alshanbari, Abdal-Aziz H. El-Bagoury

**Affiliations:** ^1^Department of Mathematics, Al-Lith University College, Umm Al-Qura University, Mecca, Saudi Arabia; ^2^Department of Mathematics, Faculty of Science, Assiut University, Assiut, Egypt; ^3^Department of Mathematical Sciences, College of Science, Princess Nourah bint Abdulrahman University, P.O. Box 84428, Riyadh 11671, Saudi Arabia; ^4^Basic Science Department, Higher Institute of Engineering and Technology, El-Mahala El-Kobra, Egypt

## Abstract

For a variety of well-known approaches, optimum predictors and estimators are determined in relation to the asymmetrical LINEX loss function. The applications of an iteratively practicable lowest mean squared error estimation of the regression disturbance variation with the LINEX loss function are discussed in this research. This loss is a symmetrical generalisation of the quadratic loss function. Whenever the LINEX loss function is applied, we additionally look at the risk performance of the feasible virtually unbiased generalised Liu estimator and practicable generalised Liu estimator. Whenever the variation *σ*^2^ is specified, we get all acceptable linear estimation in the class of linear estimation techniques, and when *σ*^2^ is undetermined, we get all acceptable linear estimation in the class of linear estimation techniques. During position transformations, the proposed Liu estimators are stable. The estimators' biases and hazards are calculated and evaluated. We utilize an asymmetrical loss function, the LINEX loss function, to calculate the actual hazards of several error variation estimators. The employment of *δ*_*P*_(*σ*), which is easy to use and maximin, is recommended in the conclusions.

## 1. Introduction

The practical applications of statistics gained new emphasis [1–4]. In this approach, we consider the following. A farmer not only needs to choose the kind of fertiliser that generates the greatest mean output from a list of ‘k' fertilisers but also needs an estimation of the mean for the fertiliser he chooses. A physician needs not only to choose the kind of drugs from a list of ‘k' distinct drugs, quantify its efficiency, and choose the more efficient one but also needs to evaluate the drug's efficiency using the similar information. See [5], for more information on this subject, including debates and applications [6]. The symmetrical quadratic loss functions have been frequently employed in assessing risk functions of certain estimators. It is worth noting that all-biased estimator research employs the mean square error (MSE) or, equally, the symmetric quadratic loss as the foundation for evaluating estimator effectiveness. The employment of symmetric loss functions are well acknowledged to be incorrect in several situations, especially when positively and negatively errors have differing effects. Varian [7] developed the asymmetric LINEX (linear exponential) loss function, which is quite valuable. Since then [8], the features of the LINEX loss function have been thoroughly explored, and various research studies on the usage of the LINEX loss function have been conducted. The loss functional is obtained by estimating the variable *θ* by $\hat{\theta }$ [9]:

(1) $$\begin{array}{c} L\left(\hat{\theta }\right)=b\left[\exp\left(a\Delta \right)-a\Delta -1\right], \end{array}$$

where $a\neq 0,b>0,\text{ and }\Delta =\hat{\theta }-\theta /\theta$ are the relative estimation errors when employing $\hat{\theta }$ to evaluate $\hat{\theta }$. Because the comparative estimation errors are independent of the unit, it is frequently utilised. We consider (without losing flexibility) that *b*=1 in this research. If overestimation is much more serious than underestimation, the value of the shape factor *a* represents the orientation of asymmetry. We assign *a* > 0(*a* < 0) if overestimation is more serious than underestimation. The degree of asymmetry is represented by the size of *a*. In the case of tiny values of $\left|a\right|,L\left(\hat{\theta }\right)=1/2ba^{2}\left(\hat{\theta }-\theta /\theta \right)$ which is equivalent to a (SEL) squared error loss. As a result, the LINEX loss function could be thought of as an asymmetric generalisation of the squared error loss function. The LINEX loss function has been evaluated by a number of researchers in several interest difficulties. For instance, see [10–14]. With the LINEX loss function, Ohtani [15] investigated the risk of the feasible generalised ridge regression (FGRR) estimation. Whenever *a* is large and positive, Ohtani [16] demonstrated that the FGRR estimator could completely outperform the ordinary least squares (OLS) estimator. Using the asymmetric LINEX loss function, Wan [17] investigates the characteristics of the feasible almost unbiased generalised ridge regression (FAUGRR) estimator. Positive estimation error is considered more significant than negative estimation mistake if the variable *a* is positive, and vice versa. When multicollinearity is a challenge, one option is to employ the Liu estimators suggested by [18] (also, see [19]). Undefined variables are the finest biasing variables to use; they can be substituted by sampling estimations. The Liu estimators are referred to as viable Liu estimators in this circumstance. Akdeniz and Kaçiranlar [19] calculated the accurate MSE of the viable generalised Liu estimator. Since the usage of symmetrical loss functions might be problematic in certain practical scenarios, asymmetric loss function estimating difficulties has recently received a lot of emphasis (see, for example, [8]). The accompanying important asymmetric LINEX loss function was developed by Varian [7]:

(2) $$\begin{array}{c} L\left(\delta ,\theta \right)=b\left(\exp\left\{a\left(\delta -\theta \right)\right\}-a\left(\delta -\theta \right)-1\right), \end{array}$$

where the variables *a* ≠ 0, *b* > 0 are well-known. Using the above loss function, Zellner [8] [20] established that the ordinary sample mean is unacceptable for predicting standard mean (in the situation where the variation is available). Roio [21] extended Zellner's findings by considering the acceptability of linear functions of the sample mean under the LINEX loss function (2). Bolfarine [22] looked at estimate difficulties for the limited populations total using the LINEX loss function at the time, *θ*, in (2), meant populations' total. He presented the populations' overall Bayes estimation technique and addressed the acceptability of certain generated estimators. The goal of this study is to see if linear estimators of an independent linear function of limited population's feature variables are admissible under the LINEX loss function. Assume that the limited populations {*Y*_1_,…, *Y*_*N*_} are a random sample drawn from the superpopulations' prototype [23]:

(3) $$\begin{array}{c} y_{k}=a_{k}\beta +b_{k}+\varepsilon_{k}, \end{array}$$

where *k*=1,…, *N*, *a*_*k*_ > 0 and *b*_*k*_ were given variables, *β* is the undetermined variable, *ε*_*k*_ is standard with mean zero and variation, *σ*^2^,and *ε*_1_,…, *ε*_*N*_ are directly independent. Cassel et al. examined this concept in depth and found it to be highly beneficial. It was also addressed by [24]. Considering the superpopulation framework, we would investigate the estimation difficulties of the linear function ∑_*k*=1_^*N*^*p*_*k*_*Y*_*k*_(*p*_*k*_ > 0, *k*=1,…, *N*), with the LINEX loss function (Eq. 2 and Eq. 3). We consider that the sample {*y*_*k*_, *k* ∈ *s*} is generated using an independent sampling method *p*(*i*.*e*., *p*(*s*)satisfiesp(*s*) > 0,  and ∑_*s*∈*S*_*p*(*s*)=1, where *S* is a class of subsets of 1,…, *N*). We find all acceptable linear estimators of ∑_*k*=1_^*N*^*p*_*k*_*Y*_*k*_ in the scenario, where *σ*^2^ is given. We also analyse the acceptability of a linear estimator in this instance because *σ*^2^ is frequently undetermined in actual issues. In the class of linear estimation techniques, we achieve all acceptable linear estimation methods of ∑_*k*=1_^*N*^*p*_*k*_*Y*_*k*_. Unlike the squared error loss (SEL), the sufficient and necessary criteria for a linear estimator to be acceptable with the LINEX loss function, for scenarios where *σ*^2^ is unknown or known, are significantly varied, at least within the class of linear estimators, which is rather unexpected.

The accompanying factors are the factors why the researcher chooses linear function ∑_*k*=1_^*N*^*p*_*k*_*Y*_*k*_:

- It contains the normal situation of *E*(*ε*_*K*_^2^)=*σ*^2^*a*_*k*_^*g*^(*g* ≥ 0 is a fixed variable) through transformations
- In certain actual situations, the linear function ∑_*k*=1_^*N*^*p*_*k*_*Y*_*k*_ must be estimated [25]

We consider *b*=1 in the LINEX loss functions because the values of *b* have no effects on acceptability.

## 2. Linex Loss Functions

Zellner studied the LINEX loss functions in his research work [8]. The derivations are as discussed below. The scalar estimating errors in utilizing $\hat{\theta }$ to predict *θ* is denoted as $\Delta =\hat{\theta }-\theta$. The accompanying convex loss function was proposed by Varian [7]:

(4) $$\begin{array}{c} L\left(\Delta \right)=be^{a\Delta }-c\Delta -b,a,c\neq 0,b>0. \end{array}$$

*L*(0)=0 is clearly visible. Moreover, we need *ab*=*c* for a minimum to occur at Δ=0; therefore, (4)could be rewritten as

(5) $$\begin{array}{c} L\left(\Delta \right)=b\left[e^{a\Delta }-a\Delta -1\right],a\neq 0,b>0. \end{array}$$

In (5) there are two variables, *a* and *b*, with *b* determining the loss function's scale and *a* determining its form. For specified values of *a* and Δ, values of *e*^*a*Δ^ − *a*Δ − 1 are graphed in Figure 1. For *a*=1 or *a* > 0, it can be observed that the functions are asymmetrical, with overestimation costing more than underestimation. Whenever *a* < 0, on the contrary, (5)climbs practically exponentially when $\Delta =\hat{\theta }-\theta <0$, and approximately, linear when $\Delta =\hat{\theta }-\theta >0$.

The function is nearly symmetrical and not far from a squared error loss function for smaller values of |*a*|. Extending *e*^*a*Δ^=1+*a*Δ+*a*^2^Δ^2^/2, *L*(Δ)=*a*^2^Δ^2^/2, which is a squared error loss function. As a result, for low values of |*a*|, the best predictions and estimations are similar to those produced using a squared error loss functions. Whenever |*a*| considers significant values, meanwhile, optimum point predictions and estimations would vary significantly from those produced with a symmetrical squared error loss function; for instances, see Varian [7]. There is a desire to expand the type of estimate for multiparameter estimations and multivariate prediction challenges (4) and (5) Let $\Delta_{i}={\hat{\theta }}_{i}-\theta_{i}$ represent the errors in predicting *θ*_*i*_ with the estimate ${\hat{\theta }}_{i},i=1,2,\ldots ,k$. The separable expanded LINEX loss function is then as follows:

(6) $$\begin{array}{c} L\left(\Delta \right)=\sum_{i=1}^{k}b_{i}\left(\exp\left(a_{i}\Delta_{i}\right)-a_{i}\Delta_{i}-1\right),\\ a_{i}\neq 0,b_{i}>0,i=1,2,\ldots ,k, \end{array}$$

where Δ′=(Δ_1_, Δ_2_,…, Δ_*k*_). *L*(0)=0, *L*′(0)=0, and Δ=0 correspond to a minimum in this convex loss functions. In multiparameter multivariate prediction and estimation issues, the function in (6)could be used.

## 3. The Estimator

The estimator is discussed extensively in the research work of Parsian and Farsipour in the year 2000 who made an extensive study and derived variables, as discussed below [26]. Let *X*_*i*1_, *X*_*i*2_,…, *X*_*in*_, *i*=1,2, be a set of independent randomly sampling from standard population, each with an undetermined mean *θ*_*i*_ and a mutual determined variation *τ*^2^. Let ${\bar{X}}_{i}$ represent the sample mean of the *i*th population, where *i*=1,2. The fundamental method, according to which the population equivalent to the bigger sample mean is picked, is used to choose the population with the higher mean. We would like to calculate the population's mean *M* that could be represented as

(7) $$\begin{array}{c} M=\theta_{1}I_{1}+\theta_{2}I_{2}\\ =\theta_{2}+\theta I_{1}. \end{array}$$

Here, *θ*=*θ*_1_ − *θ*_2_, *I*_2_=1 − *I*_1_, and

(8) $$\begin{array}{c} I_{1}=\left\{\begin{array}{c} 1,\;\text{ if }{\bar{X}}_{1}.>{\bar{X}}_{2},\\ 0,\;\text{ otherwise}. \end{array}\right. \end{array}$$

*M* is, of course, a stochastic variable with a discrete property and probability functions:

(9) $$\begin{array}{c} P\left(M=\theta_{i}\right)\\ =P\left(X_{max}={\bar{X}}_{i}\right)\\ =P\left(\left\{{\bar{X}}_{i}.>{\bar{X}}_{j}.;i\neq j\right\}\right). \end{array}$$

For *i*=1,2, $X_{\text{max}}=\text{max}\left({\bar{X}}_{1}.,{\bar{X}}_{2}.\right)$.

An estimator *δ* of *θ* satisfies the preceding conditions, which are considered to be risk unbiased by [27]

(10) $$\begin{array}{c} E_{\theta }\left[L\left(\theta ,\delta \left(X\right)\right)\right],\\ E_{\theta }\left[L\left(\theta {}^{\prime },\delta \left(X\right)\right)\right],\\ \forall \theta {}^{\prime }\neq \theta . \end{array}$$

As a result, we call an estimator *δ* of *M* risk unbiased with consideration to the LINEX loss function (1) (from here on referred to as *L*-unbiased) if

(11) $$\begin{array}{c} E\left(e^{a\delta }\right)=E\left(e^{aM}\right). \end{array}$$

Otherwise, it is biased because bias is described as

(12) $$\begin{array}{c} B\left(\delta \right)=\frac{1}{a}\left\{In\left(E\left(e^{aM}\right)\right)-In\left(E\left(e^{a\delta }\right)\right)\right\}, \end{array}$$

where *M* has a normal estimation:

(13) $$\begin{array}{c} \delta_{1}=\frac{{\bar{X}}_{1}.+{\bar{X}}_{2}.}{2}+\frac{\left|{\bar{X}}_{1}.-{\bar{X}}_{2}.\right|}{2}. \end{array}$$

$X_{\max}=\max\left({\bar{X}}_{1}.,{\bar{X}}_{2}.\right)$ is unmistakable. The second estimation is generated by removing from, on its own, an *λ*-multiple of *δ*_1_'s predicted bias. This results in a slightly different class of estimators known as bias reducing (BR) estimators. They are reliant on constants *λ* that determine the degree of bias elimination and also have an impact on the hazard, which is of the type

(14) $$\begin{array}{c} \delta_{1\lambda \left(\sigma \right)}=X_{max}+\frac{a\lambda \sigma^{2}}{2}+\frac{\lambda }{a}In\left\{\frac{Ф\left(a\sigma /\sqrt{2}-X/\sqrt{2\sigma }\right)+e^{ax}Ф\left(a\sigma /\sqrt{2}+X/\sqrt{2\sigma }\right)}{1+\left(e^{aX}-1\right)Ф\left(X/\sqrt{2\sigma }\right)}\right\}. \end{array}$$

where $X={\bar{X}}_{1}.-{\bar{X}}_{2}.,\sigma =\tau /\sqrt{n},\lambda 0$ is an arbitrary variable, and *Ф*(Δ) is the usual regular overall distributions functions.

We suggest a third estimator, which is provided by

(15) $$\begin{array}{c} \delta_{3}\left(\sigma \right)={\bar{X}}_{2}.+\frac{1}{a}In\left\{1+\left(e^{aX}-1\right)Ф\left(\frac{X}{\sqrt{2\sigma }}\right)\right\}. \end{array}$$

Consider that, for a motive of (15) as an estimation of *M*, use MLE of 1/*aIn*{*E*(*e*^*aX*^)} (14):

(16) $$\begin{array}{c} E\left(e^{aM}\right)=e^{a\theta_{2}}\left\{1+\left(e^{a\theta }-1\right)Ф\left(\frac{\theta }{\sqrt{2\sigma }}\right)\right\}. \end{array}$$

This form of estimator has a broader version, which is provided by

(17) $$\begin{array}{c} \delta_{2\lambda }\left(\sigma \right)={\bar{X}}_{2}.+\frac{1}{a}In\left\{1+\left(e^{aX}-1\right)Ф\left(\frac{X}{\sqrt{2\sigma }}\right)\right\}+\frac{a\lambda \sigma^{2}}{2}\\ +\frac{\lambda }{a}In\left\{\frac{Ф\left(a\sigma /2-X/2\sigma \right)+e^{aX}Ф\left(a\sigma /2+X/2\sigma \right)}{1+\left(e^{aX}-1\right)Ф\left(X/\sqrt{2\sigma }\right)}\right\}, \end{array}$$

where *λ* is a variable. The reason for *δ*_1*λ*_(*σ*) is similar to for *δ*_2*λ*_(*σ*), and it is calculated by removing a *λ*-multiple of *δ*_3_(*σ*) estimated bias from its own. Another estimation that we will look into is provided by

(18) $$\begin{array}{c} \delta_{H}\left(c\right)=\left\{\begin{array}{c} \frac{{\bar{X}}_{1}.\;+{\bar{X}}_{2}.}{2},\;if\left|{\bar{X}}_{1}.-{\bar{X}}_{2}.\right|\sqrt{2c\sigma },\\ X_{\max},\;otherwise, \end{array}\right. \end{array}$$

where *c* is a variable that can be changed. It is worth noting that we obtain *X*_max_, for *c*=0, which is similar to *δ*_1*λ*_(*σ*) for *λ*=0. The estimator *δ*_*H*_(*c*) is frequently referred to as a hybrid estimator, and it has been taken into consideration. It is explained how *δ*_*H*_(*c*) has been adjusted. We acquire this estimator using *X*_max_ and a preliminary testing. We now develop the next estimation utilizing a concept of references. It is worth noting that, in most circumstances, the categorization of the selected group maintains to be fascinating after the decision has been made. In most cases, the preliminary decision effects are omitted in the estimation [28].

After early significant testing has been completed, the challenge of estimating arises. The post-selection estimating challenge is particularly important in the development of processes and equipment with a large number of elements, as [29] pointed out in relation to his approach. If the risk rates or another feature value of the entire system or equipment is evaluated, the accumulating bias might create quite a deceptive conclusion if both the assortments and the number of components are considerable [30].

When it comes to estimation, additional information is generally accessible than when it comes to decision. The statistics accessible at the period of choosing are denoted by *Z*_1_ and *Z*_2_, and the extra data accessible at the time of estimation are denoted by *W*_1_ and *W*_2_. *Z*_1_, *Z*_2_, *W*_1_, and *W*_2_ are clearly designed to be independent factors:

(19) $$\begin{array}{c} E\left(e^{aZ_{i}}\right)=E\left(e^{aW_{i}}\right)\\ =e^{a\theta_{i}}i\\ =1,2. \end{array}$$

This is how we characterize:

(20) $$\begin{array}{c} M_{1}=\left\{\begin{array}{c} \theta_{1},\;if\;Z_{1}Z_{2},\\ \theta_{2},\;\text{ Otherwise.} \end{array}\right. \end{array}$$

The accompanying formulas can be used to determine the parameters *Z*_*i*_ and *W*_*i*_:

(21) $$\begin{array}{c} Z_{i}={\bar{X}}_{i}.+\frac{V_{i}}{c}-\frac{1}{2}\frac{a\sigma^{2}\left(c^{2}+1\right)}{c^{2}},\\ W_{i}={\bar{X}}_{i}.-cV_{i}-\frac{1}{2}a\sigma^{2}\left(c^{2}+1\right),\;i=1,2, \end{array}$$

where *c* is a positive value and *V*_1_ and *V*_2_ are independent random factors. They are regularly generated, with a mean of 0 and a variation of *σ*^2^, and are unaffected by ${\bar{X}}_{1}.$ and ${\bar{X}}_{2}.$. They can be specified as a function of the actual sampling components or created using a table of stochastic numbers. Now, let us establish

(22) $$\begin{array}{c} U=\left\{\begin{array}{c} W_{1},\;\text{ if }Z_{1}Z_{2}\\ W_{2},\;\text{ otherwise.} \end{array}\right. \end{array}$$

It is then simple to prove that

(23) $$\begin{array}{c} E\left(e^{aM_{1}}\right)=E\left(e^{aU}\right). \end{array}$$

Specifically, *U* is an *L*-unbiased *M*_1_ estimator that is biased for *M*. Instead of *U*, a different estimate is generated as specified:

(24) $$\begin{array}{c} E\left(e^{aU}|{\bar{X}}_{1}.,{\bar{X}}_{2}.\right)=e^{a{\bar{X}}_{2}.-\left(1/2\right)a^{2}\sigma^{2}}\left[e^{aX}Ф\left(\frac{cX}{\sqrt{2\sigma }}-\frac{ac\sigma }{\sqrt{2}}\right)+Ф\left(-\frac{cX}{\sqrt{2\sigma }}-\frac{ac\sigma }{\sqrt{2}}\right)\right]. \end{array}$$

As a result, a *M* estimation is provided by

(25) $$\begin{array}{c} \delta_{4}\left(c\right)={\bar{X}}_{2}.-\frac{1}{2}a\sigma^{2}+\frac{1}{a}In\left\{e^{aX}Ф\left(\frac{cX}{\sqrt{2\sigma }}-\frac{ac\sigma }{\sqrt{2}}\right)+Ф\left(-\frac{cX}{\sqrt{2\sigma }}-\frac{ac\sigma }{\sqrt{2}}\right)\right\}. \end{array}$$

The *δ*_4_(*c*) estimator is an *L*-unbiased estimation:

(26) $$\begin{array}{c} \theta_{2}+\frac{1}{a}In\left\{\left(e^{a\theta }-1\right)Ф\left(\frac{c\theta }{\sqrt{2\sigma \sqrt{c^{2}+1}}}\right)+1\right\}, \end{array}$$

for large *c*, which becomes $\theta_{2}+1/aIn\left\{\left(e^{a\theta }-1\right)Ф\left(\theta /\sqrt{2\sigma }\right)+1\right\}$. As a result, by increasing *c*, the bias of *δ*_4_(*c*) as an *M* estimator could be reduced. The Pitman-type estimator of *M*, which is the generalised Bayesian estimation of *M* with regard to the regular priori on the two-dimensional (2D) space (*θ*_1_, *θ*_2_), is the concluding estimation under consideration:

(27) $$\begin{array}{c} \delta_{P}\left(\sigma \right)={\bar{X}}_{1}.I_{1}+{\bar{X}}_{2}.I_{2}-\frac{a\sigma^{2}}{2}I_{1}^{2}-\frac{a\sigma^{2}}{2}I_{2}^{2}. \end{array}$$

It proves to be

(28) $$\begin{array}{c} \delta_{P}\left(\sigma \right)=X_{\text{max}}-\frac{a\sigma^{2}}{2}, \end{array}$$

as well as it is a minimax.

To conclude this section, it is essential noting that whenever symmetries were available in a situation, it is normal to demand a comparable symmetry to exist for the estimation, according to the selection theoretic method. There are intrinsic symmetries in many statistics estimating issues. In our estimating issue, this is likewise the situation. The proposed estimators were stable by position modifications in the sense that if $\hat{M}$ represents for an estimator of *M*,

(29) $$\begin{array}{c} \hat{M}\left(Y_{1}+c,Y_{2}+c\right)=\hat{M}\left(Y_{1},Y_{2}\right)+c,\forall c\in R. \end{array}$$

Since *M* My1; y2 is also stable by position modifications, this is a desired characteristic.

## 4. The Feasible Gl Estimator's Risk Performance

Akdeniz widely studied the feasibility of the GL estimator risk performance [31]. According to his research work, we established a suitable requirement for the GL estimator with *d*_*i*_=⋋_*i*_(*β*_*i*_^2^ − *σ*^2^)/⋋_*i*_*β*_*i*_^2^+*σ*^2^ to dominating the OLS estimator when the LINEX loss functions are applied in the preceding section. However, in practise, this biasing factor comprises the undetermined parameters, *β*_*i*_ and *σ*^2^, that can be substituted by their sampling estimations. The practicable GL estimator has the following parameters: ${\hat{d}}_{i}=\lambda_{i}\left({\hat{\beta }}_{i}{}^{2}-{\hat{\sigma }}^{2}\right)/\lambda_{i}{\hat{\beta }}_{i}{}^{2}+{\hat{\sigma }}^{2}\text{ and }{\hat{\sigma }}^{2}={\left(y-X\hat{\beta }\right)}^{\prime }\left(y-X\hat{\beta }\right)/n-l$. In this section, we look at how the feasible GL estimator performs whenever the LINEX loss function is applied.

We'll define $z_{i}=\lambda_{i}^{2}{\hat{\beta }}_{i}/\sigma \text{ and }V=\left(n-l\right)\partial^{2}/\sigma^{2}$. Therefore, with *v*=*n* − *l* degrees of freedom, *z*_*i*_ and *V* are distributed as *N*(*θ*_*i*_, 1) and chi-square distributions, correspondingly. The feasible GL estimator of *β*_*i*_ could be expressed as using *z*_*i*_ and *V*:

(30) $$\begin{array}{c} {\tilde{\beta }}_{i}^{*}=\frac{\lambda_{i}+{\hat{d}}_{i}}{1+\lambda_{i}}{\hat{\beta }}_{i}. \end{array}$$

Or

(31) $$\begin{array}{c} {\tilde{\beta }}_{i}^{*}=\frac{\lambda_{i}+\lambda_{i}\left({\hat{\beta }}_{i}^{2}-{\hat{\sigma }}^{2}\right)/\lambda_{i}{\hat{\beta }}_{i}^{2}+{\hat{\sigma }}^{2}}{1+\lambda_{i}}{\hat{\beta }}_{i},\\ \frac{z_{i}^{2}}{z_{i}^{2}+v/\nu }{\hat{\beta }}_{i}. \end{array}$$

We can define ${\hat{\beta }}_{i}=z_{i}\beta_{i}/\theta_{i}$ since $z_{i}=\lambda_{i}^{1/2}{\hat{\beta }}_{i}/\sigma an\;d\theta_{i}=\lambda_{i}^{1/2}\beta_{i}/\sigma$. As a result,

(32) $$\begin{array}{c} {\tilde{\beta }}_{i}^{*}=\frac{z_{i}^{3}\beta_{i}/\theta_{i}}{z_{i}^{2}+v/\nu }. \end{array}$$

Or

(33) $$\begin{array}{c} \frac{{\tilde{\beta }}_{i}^{*}}{\beta_{i}}=\frac{z_{i}^{3}\beta_{i}/\theta_{i}}{z_{i}^{2}+v/\nu }. \end{array}$$

The hazard function of ${\tilde{\beta }}_{i}^{*}$ is

(34) $$\begin{array}{c} R\left({\tilde{\beta }}_{i}^{*}\right)=E\left\{\exp\left[a\left(\frac{{\tilde{\beta }}_{i}^{*}}{\beta_{i}}-1\right)\right]-a\left(\frac{{\tilde{\beta }}_{i}^{*}}{\beta_{i}}-1\right)-1\right\}\\ =E\left[\overset{\infty }{\underset{j=0}{\sum }}a^{j}\frac{{\left({\tilde{\beta }}_{i}^{*}/\beta_{i}-1\right)}^{j}}{j^{!}}\right]-E\left[a\left(\frac{{\tilde{\beta }}_{i}^{*}}{\beta_{i}}-1\right)+1\right]\\ =E\left[1+\frac{a\left({\tilde{\beta }}_{i}^{*}/\beta_{i}-1\right)}{1!}\right]+E\left[\overset{\infty }{\underset{j=2}{\sum }}a^{j}\frac{{\left({\tilde{\beta }}_{i}^{*}/\beta_{i}-1\right)}^{j}}{j^{!}}\right]-E\left[a\left(\frac{{\tilde{\beta }}_{i}^{*}}{\beta_{i}}-1\right)+1\right]\\ =E\left[\overset{\infty }{\underset{j=2}{\sum }}\frac{a^{j}}{j!}\overset{j}{\underset{r=0}{\sum }}C\left(j,\;r\right){\left(\frac{{\tilde{\beta }}_{i}^{*}}{\beta_{i}}\right)}^{r}{\left(-1\right)}^{j-r}\right]\\ =\overset{\infty }{\underset{j=2}{\sum }}a^{j}\overset{j}{\underset{r=0}{\sum }}\frac{j!}{r!\left(j-r\right)!j!}{\left(-1\right)}^{j-r}E\left[{\left(\frac{{\tilde{\beta }}_{i}^{*}}{\beta_{i}}\right)}^{r}\right]. \end{array}$$

As a result, the risk function for ${\tilde{\beta }}_{i}^{*}$ is

(35) $$\begin{array}{c} R\left({\tilde{\beta }}_{i}^{*}\right)=\overset{\infty }{\underset{j=2}{\sum }}a^{j}\overset{j}{\underset{r=0}{\sum }}\frac{j!}{r!\left(j-r\right)!j!}{\left(-1\right)}^{j-r}E\left[\frac{z_{i}^{3r}}{\theta_{i}^{r}{\left(z_{i}^{2}+v/\nu \right)}^{r}}\right]. \end{array}$$

As a result, the risk functional of the practicable GL estimator, ${\tilde{\beta }}_{i}^{*}$, satisfies the risk component of the feasible GRR estimation method, which is provided. By replacing *β*_*i*_^2^and *σ*^2^ with their unbiased estimations ${\hat{\beta }}_{i}^{2}-\partial^{2}/\lambda_{i}\text{ and }{\hat{\sigma }}^{2}$, we get the following estimates of $d_{i}:{\tilde{d}}_{i}=1-{\hat{\sigma }}^{2}1+\lambda_{i}/\lambda_{i}{\hat{\beta }}_{i}^{2},i=1,2,\ldots ,l$ (refer, for instance, Liu (1993)) [23]. The viable GL estimation of *β*_*i*_ in this example is expressed as

(36) $$\begin{array}{c} {\tilde{b}}_{i}=\frac{\lambda_{i}+{\tilde{d}}_{i}}{1+\lambda_{i}}{\hat{\beta }}_{i}. \end{array}$$

Or

(37) $$\begin{array}{c} {\tilde{b}}_{i}=\left(1-\frac{V}{vz_{i}^{2}}\right)\frac{z_{i}\beta_{i}}{\theta_{i}}. \end{array}$$

As a result,

(38) $$\begin{array}{c} \frac{{\tilde{b}}_{i}}{\beta_{i}}=\left(1-\frac{V}{vz_{i}^{2}}\right)\frac{z_{i}}{\theta_{i}}. \end{array}$$

The ${\tilde{b}}_{i}$ risk function is

(39) $$\begin{array}{c} R\left({\tilde{b}}_{i}\right)=\overset{\infty }{\underset{j=2}{\sum }}a^{j}\overset{j}{\underset{r=0}{\sum }}\frac{j!}{r!\left(j-r\right)!j!}{\left(-1\right)}^{j-r}E\left[{\left(\frac{{\tilde{b}}_{i}}{\beta_{i}}\right)}^{r}\right]. \end{array}$$

Or

(40) $$\begin{array}{c} R\left({\tilde{b}}_{i}\right)=\overset{\infty }{\underset{j=2}{\sum }}a^{j}\overset{j}{\underset{r=0}{\sum }}\frac{j!}{r!\left(j-r\right)!j!}{\left(-1\right)}^{j-r}E\left[{\left(1-\frac{V}{vz_{i}^{2}}\right)}^{r}{\left(\frac{z_{i}}{\theta_{i}}\right)}^{r}\right]. \end{array}$$

The *r*th moment of ${\tilde{b}}_{i}/\beta_{i}$ is provided as indicated in Appendix.

(a) *r*=2*p*:

(41) $$\begin{array}{c} E{\left(\frac{{\tilde{b}}_{i}}{\beta_{i}}\right)}^{2p}={\left(\frac{\theta_{i}^{2}}{2}\right)}^{-p}\overset{\infty }{\underset{q=0}{\sum }}{\left(\frac{\theta_{i}^{2}}{2}\right)}^{q}\exp\left(-\frac{\theta_{i}^{2}}{2}\right)\frac{\Gamma \left(p+q+v+1/2\right)}{q!\Gamma \left(q+1/2\right)\Gamma \left(\nu /2\right)}\\ \times \overset{1}{\underset{0}{\int }}f^{q-p-\frac{1}{2}}{\left[\frac{f\left(v+1\right)-1}{v}\right]}^{2p}{\left(1-f\right)}^{v/2-1}df. \end{array}$$

(b) *r*=2*p*+1:

(42) $$\begin{array}{c} E{\left(\frac{{\tilde{b}}_{i}}{\beta_{i}}\right)}^{2p+1}={\left(\frac{\theta_{i}^{2}}{2}\right)}^{-p}\overset{\infty }{\underset{q=0}{\sum }}{\left(\frac{\theta_{i}^{2}}{2}\right)}^{q}\exp\left(-\frac{\theta_{i}^{2}}{2}\right)\frac{\Gamma \left(p+q+v+1/2+1\right)}{q!\Gamma \left(q+3/2\right)\Gamma \left(\nu /2\right)}\\ \times \overset{1}{\underset{0}{\int }}f^{q-p-\frac{1}{2}}{\left[\frac{f\left(\nu +1\right)-1}{\nu }\right]}^{2p+1}{\left(1-f\right)}^{v/2-1}df. \end{array}$$

By replacing for (42) and (43) in (39) the risk functions could be derived.

## 5. Risk Functions

Kazhuhiro Ohtani is one of the researchers who studied the extensive risk functions involved in LINEX functions. According to him, the following discussion is done [16]. In his study, the following variables are defined first:

(43) $$\begin{array}{c} u=n\frac{{\left(\bar{x}-\mu_{0}\right)}^{2}}{\sigma^{2}},\\ v=\overset{n}{\underset{i=1}{\sum }}\frac{{\left(x_{i}-\bar{x}\right)}^{2}}{\sigma^{2}}. \end{array}$$

While *u* is allocated as *X*_1_^'2^(*λ*), *v* is allocated as *X*_*n*−1_^2^, *X*_1_^'2^(*λ*) the noncentral chi-square distributions with 1 degree of freedom, *X*_*n*−1_^2^ signifies the chi-square [31] allocation with *n* − 1 degrees of freedom, and noncentrality variable is *λ*=*n*(*μ* − *μ*_0_)^2^/*σ*^2^ Taking into account that ∑_*i*=1_^*n*^(*x*_*i*_ − *μ*_0_)^2^=*σ*^2^(*v*+*u*) and *J*=*σ*^2^*v*/*σ*_0_^2^=*v*/*θ*, wherein $\theta =\sigma_{0}^{2}/\sigma^{2}\leq 1,{\hat{\sigma }}^{*2}/\sigma^{2}$:

(44) $$\begin{array}{c} \frac{{\hat{\sigma }}^{*2}}{\sigma^{2}}=I\left(\frac{v}{\theta }<c\right)\theta +\frac{I\left(v/\theta \geq c,v/v+u<a_{1}/a_{2}\right)v}{a_{1}}\\ +\frac{I\left(v/\theta \geq c,v/v+u\geq a_{1}/a_{2}\right)\left(v+u\right)}{a_{2}}. \end{array}$$

Here, *a*_1_=*n*+1 and *a*_2_=*n*+2.

Equate

(45) $$\begin{array}{c} \exp\left(a\Delta \right)=\overset{\infty }{\underset{k=0}{\sum }}\frac{{\left(a\Delta \right)}^{k}}{k!}. \end{array}$$

The risk function of ${\hat{\sigma }}^{*2}$ with the LINEX loss is given:

(46) $$\begin{array}{c} R\left({\hat{\sigma }}^{*2}\right)=E\left[L\left({\hat{\sigma }}^{*2}\right)\right]\\ =E\left[\overset{\infty }{\underset{K=2}{\sum }}\left(\frac{a^{k}}{k!}\right){\left(\frac{{\hat{\sigma }}^{*2}}{\sigma^{2}}-1\right)}^{k}\right]. \end{array}$$

$R\left({\hat{\sigma }}^{*2}\right)$ is reduced to utilizing the binomial expansions:

(47) $$\begin{array}{c} R\left({\hat{\sigma }}^{*2}\right)=\overset{\infty }{\underset{k=2}{\sum }}\left(\frac{a^{k}}{k!}\right)\overset{k}{\underset{m=0}{\sum }}kC_{m}E\left[{\left(\frac{{\hat{\sigma }}^{*2}}{\sigma^{2}}\right)}^{m}\right]{\left(-1\right)}^{k-m}\\ \overset{\infty }{\underset{k=2}{\sum }}a^{k}\overset{k}{\underset{m=0}{\sum }}\frac{{\left(-1\right)}^{k-m}}{m!\left(k-m\right)!}E\left[{\left(\frac{{\hat{\sigma }}^{*2}}{\sigma^{2}}\right)}^{m}\right]. \end{array}$$

The standard equation for the components of the PTSV estimation $\left(i.e.,E\left[{\left({\hat{\sigma }}^{*2}/\sigma^{2}\right)}^{m}\right]\right)$ is provided in Appendix:

(48) $$\begin{array}{c} E\left[{\left(\frac{{\hat{\sigma }}^{*2}}{\sigma^{2}}\right)}^{m}\right]=\theta^{m}P\left(\frac{v}{2},\frac{\theta c}{2}\right)\\ +\frac{1}{a_{1}^{m}}\overset{\infty }{\underset{i=0}{\sum }}\omega_{i}\left(\lambda \right)\frac{2^{m}\Gamma \left(v/2+m\right)}{\Gamma \left(v/2\right)}\left[1-P\left(\frac{v}{2}+m,\frac{\theta c}{2}\right)\right]\\ -\frac{1}{a_{1}^{m}}\overset{\infty }{\underset{i=0}{\sum }}\overset{\infty }{\underset{j=0}{\sum }}\omega_{i}\left(\lambda \right)\frac{{\left(-1\right)}^{j}2^{m}}{j!\left(1/2+i+j\right)a_{1}^{1/2+i+j}}\\ \times \frac{\Gamma \left(\nu +1/2+m+i+j\right)}{\Gamma \left(\nu /2\right)\Gamma \left(1/2+i\right)}\\ \times \left[1-P\left(\frac{\left(v+1\right)}{2}+m+i+j,\frac{\theta c}{2}\right)\right]\\ +\frac{1}{a_{2}^{m}}\overset{\infty }{\underset{i=0}{\sum }}\omega_{i}\left(\lambda \right)\frac{2^{m}}{\Gamma \left(v/2\right)\Gamma \left(1/2+i\right)}\overset{m}{\underset{r=0}{\sum }}mC_{r}\\ \times \overset{\infty }{\underset{j=0}{\sum }}\frac{{\left(-1\right)}^{j}\Gamma \left(v+1/2+m+i+j\right)}{j!\left(1/2+i+m-r+j\right)a_{1}^{1/2+i+m-r+j}}\\ \times \left[1-P\left(\frac{v+1}{2}+m+i+j,\frac{\theta c}{2}\right)\right]. \end{array}$$

Here,

(49) $$\begin{array}{c} w_{i}\left(\lambda \right)=\;\exp^{i}\frac{\left(-\lambda /2\right)\left(\lambda /2\right)}{i!}. \end{array}$$

The incomplete gamma functions ratio is denoted as *P*(∝, *y*):

(50) $$\begin{array}{c} P\left(\propto ,y\right)=\frac{1}{\Gamma \left(\propto \right)}\int_{0}^{y}t^{\propto -I}\exp\left(-t\right)dt. \end{array}$$

We get the risk function equation by equating (48)into (46)

## 6. The Liu Estimator's Probability Shrinking Factor Distributions

According to Akdeniz and Öztürk, the Liu estimator probability shrinking factor and distributions were discussed as shown below [32]. Using the CLRM requirements, we need to get the density functions of ${\hat{d}}_{i}\left(i=1,2,\ldots ,p\right)$, as described in (51) [32, 33]. The accompanying theory expresses the conclusion. The Liu estimator's probability shrinking factor distributions are

(51) $$\begin{array}{c} {\hat{d}}_{i}={\hat{d}}_{i\left(OLS\right)}=\frac{\lambda_{i}\left({\hat{\beta }}_{i}^{2}-{\hat{\sigma }}^{2}\right)}{\lambda_{i}{\hat{\beta }}_{i}^{2}+{\hat{\sigma }}^{2}}, \end{array}$$

(52) $$\begin{array}{c} y=Z\gamma +\varepsilon , \end{array}$$

(53) $$\begin{array}{c} \varepsilon ∼N\left(0,\sigma^{2}I\right). \end{array}$$

**Theorem 6 .**

The density functions of ${\hat{d}}_{i\left(OLS\right)}=\lambda_{i}\left({\hat{\beta }}_{i}^{2}-{\hat{\sigma }}^{2}\right)/\lambda_{i}{\hat{\beta }}_{i}^{2}+{\hat{\sigma }}^{2}$ with the assumptions provided in (52) and (53) are provided by

(54) fd^i=e−θi/2vv/21+λi/1−d^i−1−1/21+λi/1−d^i2Γv/2v−1+1+λi/1−d^iv+1/2×∑j=0∞θi/21+λi/1−d^i−1v−1+1+λi/1−d^ij×Γv+1/2+jΓj+1Γj+1/2,

where *θ*_*i*_=*λ*_*i*_*β*_*i*_^2^/*σ*^2^and*v*=*n* − *p*.

**Proof**

From (53),

(55) $$\begin{array}{c} {\hat{d}}_{i}=\frac{\lambda_{i}\left({\hat{\beta }}_{i}^{2}-{\hat{\sigma }}^{2}\right)}{\lambda_{i}{\hat{\beta }}_{i}^{2}+{\hat{\sigma }}^{2}}\\ =\frac{v\delta_{i}-u\lambda_{i}}{v\delta_{i}+u}. \end{array}$$

where $u=v^{{\hat{\sigma }}^{2}}/\sigma^{2}∼X_{v}^{2}$ is a central Chi-square allocation with *v* degrees of freedom and $\delta_{i}={\left({\hat{\beta }}_{i}/\sigma /\sqrt{\lambda_{i}}\right)}^{2}∼X_{1}^{2}{\left(\theta \right)}_{i}$ is a noncentral Chi-square allocation with one degree of freedom and noncentrality factor *θ*_*i*_. Because ${\hat{\sigma }}^{2}$ and ${\hat{\beta }}_{i}$ are unrelated, it proves that

(56) $$\begin{array}{c} w=\frac{\delta_{i}/1}{u/v}=\lambda_{i}\frac{{\hat{\beta }}_{i}^{2}}{{\hat{\sigma }}^{2}}∼F_{\left(1,v\right)}\left(\theta_{i},0\right). \end{array}$$

With regard to density,

(57) $$\begin{array}{c} f\left(w\right)=\frac{e^{-\theta_{i}/2v\nu /2w^{-1/2}}}{B\left(1/2,v/2\right){\left(v+w\right)}^{v+1/2}}\\ \times \overset{\infty }{\underset{j=1}{\sum }}\left(\frac{\theta_{i}w/2}{v+w}\right)\frac{\Gamma \left(v+1/2+j\right)\Gamma \left(1/2\right)}{\Gamma \left(j+1\right)\Gamma \left(j+1/2\right)\Gamma \left(v+1/2\right)}w>0, \end{array}$$

where Γ(∝)=∫_0_^*∞*^*t*^∝−1^*e*^−*t*^*dt* and *B*(∝, *β*)=Γ(*α*)Γ(*β*)/Γ(∝+*β*). After that, there is the stochastic factor:

(58) $$\begin{array}{c} {\hat{d}}_{i}=\frac{v\delta_{i}-u\lambda_{i}}{v\delta_{i}+u}=1-\frac{1+\lambda_{i}}{1+w}. \end{array}$$

When using the reverse transformations,

(59) $$\begin{array}{c} w=\frac{1+\lambda_{i}}{1-{\hat{d}}_{i}}-1. \end{array}$$

possesses the density

(60) $$\begin{array}{c} f\left({\hat{d}}_{i}\right)=\frac{e^{-\theta_{i}/2vv/2{\left(1+\lambda_{i}/1-{\hat{d}}_{i}-1\right)}^{-1/2}1+\lambda_{i}/{\left(1-{\hat{d}}_{i}\right)}^{2}}}{\Gamma \left(v/2\right){\left[v-1+1+\lambda_{i}/1-{\hat{d}}_{i}\right]}^{v+1/2}}\times \overset{\infty }{\underset{j=0}{\sum }}{\left[\frac{\theta_{i}/2\left(1+\lambda_{i}/1-{\hat{d}}_{i}-1\right)}{\left(v-1+1+\lambda_{i}/1-{\hat{d}}_{i}\right)}\right]}^{j}\times \frac{\Gamma \left(v+1/2+j\right)}{\Gamma \left(j+1\right)\Gamma \left(j+1/2\right)}, \end{array}$$

with the given $-\lambda_{i}<{\hat{d}}_{i}<1$.

The density of ${\hat{d}}_{i}$ is determined by the values of *v*=*n* − *p*, *θ*_*i*_=*λ*_*i*_*β*_*i*_^2^/*σ*^2^,and *λ*_*i*_. The density functions plots are shown in Figure 2 (*forλ*_*i*_=1.5, 2,10; *σ*^2^=4; *β*_*i*_=1; *v*=20), Figure 3 (*forλ*_*i*_=15,25,35; *σ*^2^=4; *β*_*i*_=1; *v*=20), and Figure 4 (*forλ*_*i*_=55,80,100; *σ*^2^=4; *β*_*i*_=1; *v*=20), in which the values of ${\hat{d}}_{i}$ were on the horizontal axes and $f\left({\hat{d}}_{i}\right)$.

## 7. Conclusion

Under the conditions of multicollinearity, certain biased estimators, such as the Ridge and Liu types, might be able to handle the OLS estimator's drawbacks. The efficiency of the Liu estimators addressed in this research was evaluated using the asymmetrical LINEX loss function. As a result, we can determine that these Liu estimator categories are gradually equivalent. Furthermore, the LINEX loss function is more complex to estimate and implement, whereas the density function of the shrinkage biasing variables of the generalised Liu-type estimator. The characteristics of the resultant Liu estimator are probably to be affected by the random behaviour of the predicted shrinkage biasing variables. The Liu-type estimator is based on the values of *v*=*n* − *p*, *θ*_*i*_=*λ*_*i*_*β*_*i*_^2^/*σ*^2^,and *λ*_*i*_. That could be considered a variation of the Liu estimator, which is simpler to compute and implement.

## Figures and Tables

**Figure 1:** For specified values of **a**, plots of **e**^**a**Δ^ − **a**Δ − 1.

**Figure 2:** The density functional measures of ${\hat{d}}_{i}$'s graph.

**Figure 3:** The density functional measures of ${\hat{d}}_{i}$'s graph.

**Figure 4:** The density functional measures of ${\hat{d}}_{i}$'s graph.

## Data Availability

The data used to support the findings of the study are available from the corresponding author upon request.
